The article "Causes and Preventive Measures of Sports Injuries in Physical Fitness Tests in Colleges and Universities Based on Biological Characteristics" was retracted in 2023. Reasons: signs of a paper mill; suspected computer-generated content; unreliable results or conclusions; lack of ethics approval or compliance.

# Causes and Preventive Measures of Sports Injuries in Physical Fitness Tests in Colleges and Universities Based on Biological Characteristics

**DOI:** 10.1155/2021/2280205

**Published:** 2021-11-11

**Authors:** Feng Wang

**Affiliations:** School of Physical Education, Wuhan Business University, Wuhan 430056, Hubei, China

## Abstract

Biological characteristics refer to the morphological and physiological characteristics exhibited by individual organisms. The indicators of individual biological characteristics mainly include physical indicators such as height, weight, chest circumference, and health-related physical indicators such as blood pressure, grip strength, and vital capacity. This article mainly introduces the cause analysis and preventive measures of a physical fitness test in colleges and universities based on biological characteristics and intends to provide ideas and directions for the cause analysis and preventive measures of a physical fitness test in colleges and universities. This paper proposes a research method for the cause analysis and preventive measures of sports injuries in college physical fitness tests based on biological characteristics. Research experiments on the cause analysis and preventive measures of sports injuries in the physical fitness test of colleges and universities. The experimental results in this paper show that the most frequent cause of sports injuries among boys is lack of self-protection awareness, with a probability of 24.24%; among girls, the most frequent cause of sports injuries is insufficient flexibility, with a probability of 22.86%.

## 1. Introduction

Sports injury refers to the anatomical destruction or physiological disorder of human tissues or organs in sports, which is called sports injury. Its occurrence is closely related to sports training, sports technology, sports events, sports environment, and equipment, and so on. According to the time of sports injury, it can be divided into new injuries and old injuries; according to the course of the disease, it can be divided into acute injury and chronic injury (including strain and old injuries). If the prevention of sports injuries is not emphasized during the physical fitness test and corresponding preventive measures are not taken, sports injury events are likely to occur, causing physical pain and psychological pain to students. The burden on students will affect the normal study and life of students.

In sports injuries, prevention is better than cure. Therefore, in the physical process, they must first pay attention to prevention and implement the precautionary principle, as long as we have a full understanding of the importance of sports injury prevention, and conduct serious investigations and studies. Collecting lessons, mastering the law of sports injuries, and taking effective safety measures can ensure the health of students and the normal conduct of physical fitness tests in colleges and universities.

The article "Causes and Preventive Measures of Sports Injuries in Physical Fitness Tests in Colleges and Universities Based on Biological Characteristics" was retracted in 2023. Reasons: signs of a paper mill; suspected computer-generated content; unreliable results or conclusions; lack of ethics approval or compliance.

Oppewal and Hilgenkamp proposed a set of basic physical fitness tests that can be used for young people, including physical appearance, muscle strength, muscle endurance, and balance tests. Oppewal and Hilgenkamp's recommendations for future research include extending the research to more psychometric characteristics of adaptive testing and combining the population's physical fitness data in a larger data set. This study lacks experimental data support [1]. Meshizuka and Nakanishi believed that in addition to young athletes in Japan, attention to the physical health of people of all ages is also increasing year by year. To show their actual physical fitness, Meshizuka and Nakanishi planned to conduct a set of research experiments on physical fitness tests, but it is not easy to obtain suitable test items, supplemented by scientific and accurate specifications to assess and diagnose the level of physical health. The purpose of the research is to collect as many basic data samples as possible for people of all ages. These simple physical test items are standardized. This study has not been tested in actuality and has no reference [2]. Lemos et al. studied the correlation between physical measurement parameters of female hockey players with and without the ball, Sargent jump test, core muscle endurance and agility, and specific tests. Nine professional female hockey players (age: 27.4 ± 2.5 years old) participated in this study. The authors tested their height, weight, and body fat percentage and performed the Sargent jump test (SJT), shuttle flexibility test (SR), core muscle endurance test, exercise specific test, and repeated sprint test (RSA), and the test sequence adopts the random sampling method. Results: There was a moderate correlation between SR and RSAB (*r* = 0.58; *p*=0.09) and RSA (*r* = 0.60; *p*=0.08). This research is not practical [3].

The innovations of this paper are: (1) proposed a decision tree-based college physical fitness test for sports injury data mining collection, (2) proposed ridge regression analysis method, and (3) designed a college physical fitness test system based on biological characteristics. This paper explores the sports injury parts, injury types, and injury occasions of college students majoring in physical education, as well as the influencing factors on the incidence of sports injury of college students majoring in physical education. Thus, it provides a good reference for the development of sports.

The article "Causes and Preventive Measures of Sports Injuries in Physical Fitness Tests in Colleges and Universities Based on Biological Characteristics" was retracted in 2023. Reasons: signs of a paper mill; suspected computer-generated content; unreliable results or conclusions; lack of ethics approval or compliance.

## 2. Methods of Reason and Preventive Measures for Sports Injuries in Physical Fitness Tests in Colleges and Universities Based on Biological Characteristics

### 2.1. Review on the Research of Sports Injury Theory

In daily sports, soft tissue injuries are widespread and divided into two categories: open soft tissue injuries and closed soft tissue injuries [4]. The symptoms and prevention of closed soft tissue injuries are relatively difficult. After various events, sports injuries are its regularity and clinical manifestations, such as most football players with acute head contusion; long-distance runners are more prone to fatigue periostitis; the thrower's shoulders, elbows, waist muscles, ligaments, and fascia will be strained [5]. An acute injury can usually be observed with muscle, tendons, ligament, and cartilage injury. The pressure of bone tissue, nerve tissue, and cardiovascular system is mostly caused by chronic injury or multiple small injuries, increasing the incidence of acute injury [6].

Acute sports injuries are generally caused by one-time damage caused by a large force. It usually has a rapid onset, short course, obvious pathological changes, and obvious symptoms [7]. Generally, its pathological manifestations are rapid swelling of local tissues, blood stasis, congestion accompanied by strong pain, dysfunction or loss, and mental changes (such as syncope, coma, shock, etc.) [8]. The symptoms of acute sports injury are local swelling of the injured part, red surroundings, reddish-purple, unbearable pain, tenderness, and swelling [9]. Anyone whose partial or overall dysfunction has not disappeared after the injury is forbidden to manipulate the injured part at will [10].

Some of the causes of chronic injuries are due to improper treatment of acute injuries, and some are caused by local long-term overburden, which causes continuous strain on the tissues and gradually accumulates in minor injuries [11]. Long-term repetition of a fixed action under fatigue can also cause chronic injury. The general pathological manifestations are due to local long-term excessive load, resulting in neuromodulation dysfunction, the internal synthesis and decomposition balance of the tissue is out of balance, and the structure of sugar, lipids, and proteins in the tissue is changed or even destroyed [12]. Tissue cell dystrophy, lipid changes, and fibrous tissue hyperplasia will seriously affect blood circulation, cause local Qi and blood deficiency, and even produce thrombus. The flow of Qi and blood is blocked, causing local tissue necrosis [13]. The symptoms of chronic tissue injury are insidious, with slight swelling and congestion of local tissues and slight dysfunction. In the beginning, there are local feelings of acid, numbness, and swelling; then poor elasticity, induration, local hardening and thickening, aggravation of acid, numbness, swelling, and pain; and later the pain intensification, local coldness, hindered activity, and hypofunction, and so on [14]. Chronic injury is a sports injury caused by various tissues and organs of the body after repeated lighter external forces or due to delays in curing after minor acute injuries [15].

The article "Causes and Preventive Measures of Sports Injuries in Physical Fitness Tests in Colleges and Universities Based on Biological Characteristics" was retracted in 2023. Reasons: signs of a paper mill; suspected computer-generated content; unreliable results or conclusions; lack of ethics approval or compliance.

### 2.2. Smart Healthcare

In the past two years, smartphones and mobile healthcare have opened up many new entrepreneurial opportunities and application scenarios. All kinds of new players are rushing in. They are mainly divided into B2B models for hospitals and doctors and B2C models directly for users. The former is considered professional. People mainly provide medical knowledge, while the latter is a “self-examination + consultation” telemedicine health consultation application. The advent of smart hospital applications not only can simplify the medical treatment process and reduce medical costs but also can increase the feeling of being valued by doctors; for doctors, it not only can reduce labor time but also can improve the quality of patient management and improve the level of diagnosis and treatment. For the hospital, it can more directly understand the needs of patients, serve them, improve service satisfaction, and build a harmonious doctor-patient relationship.

### 2.3. Data Mining and Collection of Sports Injuries in College Physical Fitness Tests Based on Decision Trees

Nowadays, the application of computers and networks in schools has been very popular. Computer technology can be used to carry out simple operations such as statistical analysis and screening of students' physical test results. According to the evaluation of students' physical fitness and related test information, the results of students' physical test results can be formed evaluation model to dig out the factors behind the students' physical test scores [16]. Using data mining technology to process the results of the physical fitness test of college students, further analyze the related laws hidden behind the data, dig out the influencing factors of physical sports injuries, and then analyze and study the measures to prevent injuries [17, 18].

The most widely used algorithms in decision-making algorithms are the ID3 algorithm and the C4.5 algorithm, which use a top-down method to construct a decision tree from the training tuple set and their associated class labels. As the tree is constructed, the training set is recursively divided into smaller subsets [19]. The algorithm is a recursive algorithm that requires three parameters to call the algorithm, and the algorithm returns the root node of the constructed tree [20]. Assuming that the current node is *V*, the training data set of *V* is *L*, there are *k* different class labels *C*_*i*_(*i*=1,2,…, *k*), let *C*_*i*,*L*_ be the tuple set of a class label *C*_*i*_ in *L*, and |*L*| and |*C*_*i*,*L*_| are the number of tuples. According to a certain division method, *L* is divided into *y* subsets {*L*_1_, *L*_2_,…, *L*_*y*_}.

The article "Causes and Preventive Measures of Sports Injuries in Physical Fitness Tests in Colleges and Universities Based on Biological Characteristics" was retracted in 2023. Reasons: signs of a paper mill; suspected computer-generated content; unreliable results or conclusions; lack of ethics approval or compliance.

The information gain on a certain division attribute *N* is defined as the difference between the amount of information (entropy) needed to identify tuples before division and the amount of information needed to identify tuples after division on attribute *N* [21]. There is the following relationship:

(1) $$\begin{array}{c} \text{InfoGain}\left(N\right)=\text{Info}\left(L\right)-{\text{Info}}_{N}\left(L\right),\\ \text{Info}\left(L\right)=-\sum_{i=1}^{k}p_{i}\log_{2}\left(p_{i}\right),\\ p_{i}=P\left(t\in C_{i}|\forall t\in L\right),\\ {\text{Info}}_{N}\left(D\right)=\sum_{j=1}^{y}\frac{\left|L_{j}\right|}{\left|L\right|}\times \text{Info}\left(L_{j}\right). \end{array}$$

The information gain metric tends to use attribute partitioning with more branches, and the gain rate metric is adopted, which uses the split information value to normalize the information gain [22]. The definition formula of split information is as follows:

(2) $$\begin{array}{c} {\text{SplitInfo}}_{N}=-\sum_{j=1}^{y}\frac{\left|L_{j}\right|}{\left|L\right|}\times \;\log_{2}\left(\frac{\left|L_{j}\right|}{\left|L\right|}\right). \end{array}$$

The gain rate is defined as follows:

(3) $$\begin{array}{c} \text{GainRatio}\left(N\right)=\frac{\text{InfoGain}\left(N\right)}{\text{SplitInfo}\left(N\right)}. \end{array}$$

The Gini index is the measurement criterion used in the CART algorithm. The Gini index measures the impurity of the data partition or the training tuple set *L* [23]. Its definition formula is as follows:

(4) $$\begin{array}{c} \text{Gini}\left(L\right)=1-\sum_{i=1}^{k}p_{i}^{2},\\ p_{i}=p\left(t\in C_{i}|\forall t\in L\right). \end{array}$$

The Gini index considers the binary division of each attribute. Assuming that *L* is divided into *L*_1_ and *L*_2_ for a certain binary division of attribute *N* of *L*, the Gini index of this division is defined as follows:

(5) $$\begin{array}{c} {\text{Gini}}_{N}\left(L\right)=\frac{\left|L_{1}\right|}{\left|L\right|}\text{Gini}\left(L_{1}\right)+\frac{\left|L_{2}\right|}{\left|L\right|}\text{Gini}\left(L_{2}\right). \end{array}$$

The decrease in impurity due to this division is defined as follows:

(6) $$\begin{array}{c} \Delta \text{Gini}\left(N\right)=\text{Gini}\left(L\right)-{\text{Gini}}_{N}\left(L\right). \end{array}$$

Each time the attribute that can maximize the reduction of impurity is selected as the split attribute, this attribute and its split subset (discrete value attribute) or split point (continuous value attribute) together form a split criterion [24].

The article "Causes and Preventive Measures of Sports Injuries in Physical Fitness Tests in Colleges and Universities Based on Biological Characteristics" was retracted in 2023. Reasons: signs of a paper mill; suspected computer-generated content; unreliable results or conclusions; lack of ethics approval or compliance.

### 2.4. Ridge Regression Analysis

Take sprint, standing long jump, strength quality, and endurance quality indicators as dependent variables, with height, weight, chest circumference, sitting height, triceps skinfold thickness, subscapular skinfold thickness, vital capacity, grip strength, systolic blood pressure, and diastolic blood pressure as an independent variable for analysis [25]. Ridge regression analysis is a multiple linear regression analysis method used to deal with the problem of collinearity between variables. This method is at the cost of giving up part of the information in the independent variables, and the regression effect is slightly worse but can better reflect the actual situation [26]. Ridge regression is defined as follows:

(7) $$\begin{array}{c} \beta \left(k\right)={\left(X^{,}X+kI\right)}^{-1}X^{\prime }Y, \end{array}$$

where *k* is called the ridge parameter, which is very subjective [27]. Generally, the ridge trace method, the variance expansion factor method, and the Hoerl Kennard formula method are used to determine the *k* value [28].

Principles for determining the value of *k*: (1) As the value of *k* increases, the ridge trace curve will change. When *k* = *k*_0_, the slope of the ridge trace curve begins to stabilize, and *k*_0_ at this time is the required *k* value. (2) When using other regression analysis methods for research, the signs of some independent variables are illogical, but after using the ridge regression analysis method, the signs are logical. (3) The coefficient signs of the variables in the ridge regression equation obtained are all logical. (4) The increase of the residual sum of squares tends to stabilize [29].

Principles for the elimination of independent variables: (1) The independent variables whose standardized regression coefficients in the ridge regression equation have very small absolute values and relatively stable changes. (2) With the increase of the *k* value, the ridge trace graph shows that the regression coefficients change unstable and tend to zero independent variable variables. (3) The ridge trace plot shows the independent variables whose regression coefficients vary greatly as the value of *k* increases. Ridge regression analysis has no objective criteria for the selection of independent variables. Generally, it can be determined whether the variable should be deleted according to the ridge regression result obtained by recalculating after removing some variables [30, 31].

The article "Causes and Preventive Measures of Sports Injuries in Physical Fitness Tests in Colleges and Universities Based on Biological Characteristics" was retracted in 2023. Reasons: signs of a paper mill; suspected computer-generated content; unreliable results or conclusions; lack of ethics approval or compliance.

The method part of this article uses the above methods to study the cause analysis and preventive measures of sports injuries in college physical fitness tests based on biological characteristics. The specific process is shown in Figure 1.

## 3. Design Experiment of College Physical Fitness Test System Based on Biological Characteristics

### 3.1. Data Collection Framework Design

At present, there are corresponding physical fitness testers for the eight subjects in the physical fitness test of college students on the market. Therefore, when the system is actually deployed, the test site, such as the stadium, is divided into several test areas according to the test subjects, and the test areas are selected according to the test subjects. The physique tester is used as a wireless sensor node, and then according to the size of the test area, appropriate wireless communication means are selected, and the main controller and coordinator are deployed in appropriate positions in the test area of different subjects, which can be within the wireless communication range of all wireless sensor nodes. The data of each physical fitness tester can be transmitted to each main controller in the test area. After each main controller summarizes the data transmitted by each physical fitness tester of this subject, it is transmitted to the server through the external network. Namely, it can achieve the purpose of data collection and data transmission.

The system is mainly composed of a server, the main controller module, a wireless communication module, and a sensor node module. The server is the PC that uses the Spark computing framework for data analysis and processing; the wireless communication module is divided into communication between each sensor node and the coordinator, ZigBee communication module, and the 4G wireless transmission module for remote wireless transmission between the main controller module and the server; and the main controller module uses the STM32F103ZET6 chip and the CC2530 chip to integrate through UART serial communication and is responsible for receiving the data sent by each sensor node that contains data, which will be initially processed later and sent back to the server through the 4G network. The sensor node module is composed of sensors that sense the data and CC2530 and is responsible for collecting the physical test results of students in the detection area. All modules work together to achieve the function of data collection together.

The article "Causes and Preventive Measures of Sports Injuries in Physical Fitness Tests in Colleges and Universities Based on Biological Characteristics" was retracted in 2023. Reasons: signs of a paper mill; suspected computer-generated content; unreliable results or conclusions; lack of ethics approval or compliance.

### 3.2. Sensor Node Module Design

The sensor node module comprises a sensor module, a data processing module, and a ZigBee wireless communication module. The sensor module is a variety of sensors that can collect the required data. The data processing module and the ZigBee wireless transmission module are composed of the CC2530 chip and its auxiliary circuits. Data collection, data short-distance transmission, and other purposes are jointly completed. Since the test area is not large, ordinary wireless sensor nodes do not need to communicate with each other.

#### 3.2.1. Sensor Module Design

The design of the sensor module mainly involves the selection of sensors. The subjects involved in the “New Standard” can be classified as follows according to their measurement principles: sit-ups and pull-ups are count subjects; seated forward bends, standing long jump, and height are distance measurement subjects; 50- and 800-meter running and the 1,500-meter race are time subjects; height and vital capacity are measurement subjects.

For counting subjects, infrared sensors are used for measurement; for timing subjects, infrared sensors are also used for measurement. The transmitter of the infrared sensor will continuously emit infrared signals, and when the infrared rays touch an object, they will produce a reflected signal. After receiving the signal, the receiving end performs a series of operations on the signal, such as amplifying, detecting, and shaping. Finally, it obtains a TTL level coded signal, which is sent to the CC2530 chip for decoding and subsequent operations.

For distance testing, the ultrasonic distance measurement module is selected to achieve noncontact measurement. Its working principle is to start the timer while triggering the ranging, the transmitting module will automatically send a square wave, and the high level will last for a long time. It is the time from transmission to return of the ultrasound, and the distance to the measured object can be calculated according to the time difference between transmission and reception.

The lung capacity sensor uses the XGZP6847 gas pressure sensor for measurement. The sensor consists of an elastic membrane and four resistors integrated into the membrane. When pressure acts on the elastic membrane, the bridge will generate a linear proportional to the applied pressure.

The weight measurement adopts a resistance strain pressure sensor with a maximum range of 200 kg, which has the characteristics of high precision and a simple structure. Equipped with a load-bearing plate and a mounting base, the human body can stand on the load-bearing platform for testing, avoiding the shortcomings of weighing errors caused by changes in the working plane. Its working principle is that the external elastic body will be deformed when weighing, and the resistance strain gauge will also deform, which will affect its resistance and generate a corresponding differential signal. Therefore, in the actual measurement, the sensor converts the weight into a voltage signal and then processes the voltage signal after ADC conversion to obtain the weight data.

The article "Causes and Preventive Measures of Sports Injuries in Physical Fitness Tests in Colleges and Universities Based on Biological Characteristics" was retracted in 2023. Reasons: signs of a paper mill; suspected computer-generated content; unreliable results or conclusions; lack of ethics approval or compliance.

#### 3.2.2. Design of Wireless Sensor Node

The data processing of the wireless sensor module adopts the CC2530 wireless single-chip microcomputer chip. CC2530 is a system-level SoC chip, which combines an industrial-grade compact and efficient 8051 controller and a 2.4 GHz direct sequence spread spectrum radio frequency transceiver core, which has excellent performance RF transceiver, programmable flash memory in the system, and other powerful features, with a microprocessor module and a wireless transceiver module in one.

This text uses IAR to design the wireless sensor module and the coordinator in the main control module and uses MDK5 to design the STM32 in the main control module. Due to the star topology, the coordinator connecting the sensor module and the main controller module through serial communication adopts fixed-point transmission for networking.

### 3.3. Main Controller Module Design

#### 3.3.1. Hardware Design

This text adopts the processor chip STM32F103ZET6. This chip has higher code density, abundant register, and simple addressing mode and integrates many kinds of interfaces such as TIMER, SPI, and DMA. Therefore, it can realize ZigBee wireless transmission with the sensor module and 4G communication with the server through the UART interface using asynchronous serial communication. The coordinator in this article uses the same chip as the sensor node, that is, the CC2530 chip.

#### 3.3.2. Software Design

The communication from the coordinator to the sensor node takes the form of a broadcast. The software purpose of the coordinator is mainly to create a ZigBee network and communicate with wireless sensor nodes. After configuring the Zglobals.h file in the ZigBee protocol stack network layer file, it can be determined that the CC2530 as the coordinator is used as a coordinator in the ad hoc network. If the device exists, a ZigBee network can be created during work. After the network is established, the broadcast event will be triggered periodically according to the time set by the timer. In the physique test system, the broadcast event mainly commands the wireless sensor node to transmit data.

### 3.4. Wireless Transmission Module Design

The wireless transmission module of the external network adopts the AS01-ML01DP5 wireless transmission module. Its working frequency is 2.4 GHz; it adopts a dual in-line SMA output interface, built-in LNA, integrated RFX2401C power amplifier chip, and NRF24L01 radio frequency chip. This module uses the STM8L101F3P6 smallest system board that leads out all I/O ports to realize the interface conversion function through the CH340 virtual serial port chip. According to register configuration requirements, design communication timing to control the receiving and sending of data.

The article "Causes and Preventive Measures of Sports Injuries in Physical Fitness Tests in Colleges and Universities Based on Biological Characteristics" was retracted in 2023. Reasons: signs of a paper mill; suspected computer-generated content; unreliable results or conclusions; lack of ethics approval or compliance.

This part of the experiment proposes the above steps to be used for designing experiments of a college physical fitness test system based on biological characteristics. The specific process is shown in Table 1.

## 4. Causes and Preventive Measures of Sports Injuries in College Physical Fitness Tests Based on Biological Characteristics

### 4.1. Experiment Analysis

#### 4.1.1. Research Object

The research object is a freshman to a senior in a college of a certain university. According to the logical boundary value table of each measurement index in the “National Student Physical Fitness Survey.” There are 2,246 freshmen, 2,471 sophomores, 2,139 juniors, and 2,125 seniors, as shown in Table 2 and Figure 2.

It can be seen from the chart that the selection of research objects is relatively average, the gap between grades is small, and the gap between the number of men and women is also small, which makes the experimental data more convincing and the experimental conclusions more representative. This fully shows that although physical education students rarely have serious sports injuries such as fractures in sports, the incidence of soft tissue injuries such as contusion is still high. It is inevitable for students to have sports injuries when they are engaged in basketball sports, which requires teachers to teach students relevant recovery and prevention measures so that students can master these knowledge at the same time to improve the awareness of self-protection.

#### 4.1.2. Analysis of Sports Injuries

1. Calculate the height and weight of freshman to senior students in a college and a certain college, and plot the overweight detection rate of students by a chart, as shown in Table 3 and Figure 3.
2. It can be seen from the chart that the overweight detection rate for freshmen is the largest, 16.14% for boys and 10.47% for girls. From the overall situation of the four grades, the overweight detection rate of senior students is generally lower than that of lower grades. Among students, the detection rate of male overweight is generally higher than that of female students.
3. Number of sports injuries in the physical fitness test
4. The investigation of the incidence of sports injuries mainly includes two problems, namely the number of sports injuries that have occurred since the beginning of the physical fitness test and the number of sports injuries during the physical fitness test during college, as shown in Table 4 and Figure 4.
5. It can be seen from the chart that among the 8,981 students who received the test, 719 had not been injured in the physical fitness test, accounting for only 8.01%. From the beginning of the physical fitness test to the present, there are 3,543 students who have experienced a sports injury, accounting for 39.45%, which is the highest proportion. Totally 4,541 students have undergone a physical fitness test and have experienced a sports injury during college, accounting for 50.56%, which is the highest proportion; students with two sports injuries account for 26.77%; students with three sports injuries account for 8.18%.
6. Physical fitness test and sports injury type
7. Sports injuries are like diseases. There are many types and forms, and there are different classification methods. Commonly used sports injury classification methods are: according to the structure of the injured tissue, such as skin, joints, bones, nerves, internal organs, and muscles, injury can be divided. According to the integrity of the skin or mucous membrane after injury, it is divided into open injury and closed injury. The former has wounds that communicate with the outside world, such as abrasions, stab wounds, lacerations, and open fractures; the latter has no wounds and external connections, such as contusions, sprains, strains, and closed fractures. According to the severity of the injury, it can be divided into minor injuries, medium injuries, and severe injuries. According to the severity of the injury, it can be divided into acute injury and chronic injury. For the convenience of analysis, this article divides the types of sports injuries in college physical fitness tests into strains, sprains, bruises, and fractures. The specific situation is shown in Table 5 and Figure 5.
8. The types of sports injuries of students who have experienced physical fitness sports injuries in college are not single and uneven. It shows that the number of people with strains is the largest, accounting for 48.06% of the total number of injuries during college; the second is sprains, accounting for 41.96% of the total number of injuries.

The article "Causes and Preventive Measures of Sports Injuries in Physical Fitness Tests in Colleges and Universities Based on Biological Characteristics" was retracted in 2023. Reasons: signs of a paper mill; suspected computer-generated content; unreliable results or conclusions; lack of ethics approval or compliance.

#### 4.1.3. Data Analysis

To realize the correlation between the physical test and sports injury, the PEP-Growth algorithm is used to process the data. First, the frequent item sets are generated, and the support degree is set to obtain the frequent patterns, that is, the occurrence of a certain pattern in the established database. The number of times divided by the number of records of this type of data in the database will not be lower than the set support degree. Otherwise, it is regarded as an infrequent mode, and the appearance of this mode is considered accidental and not valuable. In the setting of support, because the fitness test data is surely highly in line with the normal distribution, if the support is set high, there will be few laws that can be unearthed. Therefore, this article tries multiple supports and then finds the rules to filter. The confidence level is set to 0.7. That is, if a frequent pattern is *X*, the probability of *X* ≥ *Y* appearing in all frequent patterns *X* is greater than 0.7, and the strong rules mined are considered reliable at this time. The specific situation is shown in Table 6.

It can be seen from Table 5 that the confidence levels of pull-ups, sprint, long-distance running, long jump, and sit-ups are all higher than 0.7, showing a strong correlation. Among them, the sprint test has the strongest correlation, with a confidence of 0.977; the sprint test, as a sport that uses instantaneous explosive power, can easily lead to muscle strain and even damage to the knee.

### 4.2. Causes of Sports Injuries

#### 4.2.1. Irregular Technical Actions

Sports injuries in college students' physical fitness tests and irregular technical movements are essential factors. The various techniques in physical fitness testing usually require the coordination of various parts of the athlete's body, and wrong technical actions can cause excessive bending and stretching of joints and muscles of the body, which violates the characteristics of human structure and functions and the mechanics of exercise principle; sports injuries are extremely prone to occur.

#### 4.2.2. Insufficient Preparation Activities

The purpose of warm-up activities is further to improve the excitability of the central nervous system, enhance the functional activities of various organ systems, and make the human body transition from a relatively static state to a tense state of activity. When the function of the nervous system and various organs of the body were not fully mobilized, the students under the test were put into intense exercise. The muscle strength, elasticity, and stretchability were relatively poor, and the body lacked the necessary coordination. That is, it is often said that the “warm-up” effect is not achieved, and sports injuries are prone to occur at this time.

#### 4.2.3. Inattention

College students are prone to inattention during the test. Inattention during training or competition can deform technical movements, increase the burden on the body, and cause sports injuries. Two factors affect students' attention: internal factors and external factors; internal factors include students' bad mood, depression, irritability, their own personality characteristics, the influence of physical illness, and too much emphasis on test results, while external factors include interference from outside people or things, testing the impact of weather and environment.

The article "Causes and Preventive Measures of Sports Injuries in Physical Fitness Tests in Colleges and Universities Based on Biological Characteristics" was retracted in 2023. Reasons: signs of a paper mill; suspected computer-generated content; unreliable results or conclusions; lack of ethics approval or compliance.

#### 4.2.4. Excessive Physical Fatigue

Before taking the test, students may take the test in a state of poor sleep or rest, illness, injury, or recovery from the injury, which can easily cause excessive physical fatigue. The manifestations of overfatigue include decreased exercise level, a significant decrease in muscle strength and physical coordination, decreased concentration, and slow response. At this time, when a higher intensity test is performed, sports injuries are prone to occur.

#### 4.2.5. Insufficient Flexibility

Flexibility in sports refers to the ability of human joints to move in different directions and the ability to stretch soft tissues such as muscles and ligaments. Flexibility is manifested by the range of joint motion, that is, the range of motion generated by a certain axis of motion. It can be said that poor flexibility is one of the most important physical factors for students' sports injuries when undergoing physical fitness tests.

#### 4.2.6. Lack of Self-Protection Awareness

There are many times when students have sports injuries because they do not pay enough attention to injury prevention, their ideological negligence, and lack of necessary prevention knowledge. In particular, college students have relatively little professional experience, often a lack of understanding of the impact of sports injuries on themselves, and a lack of experience in preventing sports injuries. They have little or no learning about sports injury prevention and rehabilitation. In addition, when physical discomfort occurs, it is difficult for college students to judge the precursors of sports injuries, so they often fail to get timely treatment and delay their illness or adopt incorrect treatment and mitigation methods to make their illness worse.

Roughly calculate the frequency of the causes of sports injuries and draw graphs, as shown in Table 7 and Figure 6.

From the chart data and calculations, it can be seen that the most frequent cause of sports injuries among boys is the lack of self-protection awareness. Among boys, the least frequent cause of sports injuries is insufficient flexibility, and the least frequent cause of sports injuries among girls is lack of self-protection.

The article "Causes and Preventive Measures of Sports Injuries in Physical Fitness Tests in Colleges and Universities Based on Biological Characteristics" was retracted in 2023. Reasons: signs of a paper mill; suspected computer-generated content; unreliable results or conclusions; lack of ethics approval or compliance.

### 4.3. Preventive Measures Analysis

#### 4.3.1. Improve Awareness of Sports Injuries

College students should ideologically improve and deepen their understanding of sports injuries, understand the importance of sports injuries in their daily lives, attach importance to sports injuries ideologically, and avoid actions that risk injury during training and self-activity, only by ideologically increasing the importance of sports injuries, avoiding unnecessary human injury factors, and reducing the occurrence of sports injuries.

#### 4.3.2. Consciously Do Relaxation Exercises after the Test

Human body function is improved based on the complete recovery of the energy materials consumed during exercise. On the contrary, excessive fatigue will occur, resulting in a decline in exercise capacity and even sports injuries. After high-intensity exercise, relaxation exercises or massage can reduce muscle stiffness, effectively reduce delayed-onset muscle soreness of skeletal muscles, help eliminate lactic acid, and accelerate functional recovery.

#### 4.3.3. Learn to Protect and Supervise Yourself

Through learning relevant theoretical knowledge, have a certain understanding and mastery of sports training and sports injuries; apply the relevant theoretical knowledge learned to daily training, study, life, and extracurricular activities; and try to achieve reactive self-protection and avoid or reduce minor sports injuries. Learn to observe and analyze changes in body function; make judgments about your physical state before, during, and after exercise; learn to detect your pulse and body reactions; and judge whether the situation during training is normal and whether you need to rest. Through the monitoring of one's own physical state, the physical state is fed back to the instructor, and the teacher's opinion is used for targeted recovery or rest.

In addition, in colleges and universities, the importance of sports injuries in physical fitness testing should be strengthened. The ideological attention to the adverse effects of injuries on students is the outstanding performance of schools putting safety first. When dealing with students who have already suffered sports injuries, it is necessary to make correct judgments and make timely decisions, arrange appropriate plans according to the students' conditions to help students recover, develop scientific and reasonable test plans, take protective measures for physical testing, and strengthen the maintenance of testing venues and equipment.

## 5. Conclusions

Sports injury is a common problem encountered in physical fitness tests. From the perspective of the occurrence, one part is related to the characteristics of the project, and the other is related to the accident. Once a sports injury occurs, it is very difficult to treat because, so far, there is no particularly effective method for injury treatment, and students are often treated while studying and living. At this time, if they are not properly arranged, new injuries will be caused. It significantly prolongs the healing time of the injury. Therefore, in a sense, preventing injury is more important than treating the injury.

The article "Causes and Preventive Measures of Sports Injuries in Physical Fitness Tests in Colleges and Universities Based on Biological Characteristics" was retracted in 2023. Reasons: signs of a paper mill; suspected computer-generated content; unreliable results or conclusions; lack of ethics approval or compliance.

College students should develop the habit of consciously abiding by the order no matter how they practice any project; enhancing the awareness of protection is to avoid injury. The prerequisite is to learn the safety protection measures in various technologies, master the operating skills of self-protection and mutual protection, and move the six major joints of the body: shoulder joint, hip joint, Knee joints, ankle joints, wrist joints, and elbow joints, as well as the neck, waist, back, legs, and proper jogging are all indispensable. The blood supply to all parts ensures that aerobic exercise is dominant.

Schools should strengthen the education of students' attention to sports injuries. Through broadcasting, publicity columns, knowledge lectures, knowledge competitions, and classroom teaching, students are strengthened to educate students on safety, organization, and discipline and attach great importance to the prevention of sports injuries so that they can fully realize the harm of sports injuries to the body and the significance of preventing injuries, strengthen protection awareness, and reduce or avoid sports injuries.

## Figures and Tables

**Figure 1:** Part of the technical flow chart of this method.

**Figure 2:** Distribution of research objects.

**Figure 3:** Detection rate of overweight students.

**Figure 4:** Number of sports injuries in the physical fitness test.

**Figure 5:** Types of sports injuries in college physical fitness tests.

**Figure 6:** Frequency of causes of sports injuries.

**Table 1:** The experimental procedure of this article.

Design experiment of college physical fitness test system based on biological characteristics	Data collection framework design	College physical test system	
	Sensor node module design	1	Sensor module design
		2	Wireless sensor node design
	Main controller module design	1	Hardware design
		2	Software design
	Wireless transmission module design	AS01-ML01DP5	

**Table 2:** Distribution of research objects.

Grade	Total number of people	Number of boys	Number of girls
Freshman	2,246	1,171	1,075
Sophomore	2,471	1,230	1,241
Junior	2,139	1,064	1,075
Senior year	2,125	991	1,134

The article "Causes and Preventive Measures of Sports Injuries in Physical Fitness Tests in Colleges and Universities Based on Biological Characteristics" was retracted in 2023. Reasons: signs of a paper mill; suspected computer-generated content; unreliable results or conclusions; lack of ethics approval or compliance.

**Table 3:** The overweight detection rate of students.

Grade	Percentage	
Freshman	Boys	16.14%
	Girls	10.47%

Sophomore	Boys	15.17%
	Girls	9.35%

Junior	Boys	14.46%
	Girls	9.74%

Senior year	Boys	14.96%
	Girls	9.71%

**Table 4:** Physical fitness test and sports injuries.

Options		Zero times	Once	Twice	Three times	Four times	Above four times
From the beginning of the physical test to the present	Number of boys	382	1,726	1,344	456	296	252
	Number of girls	337	1,817	1,481	591	184	115
	Percentage	8.01%	39.45%	31.45%	11.66%	5.34%	4.09%

During college	Number of boys	382	2,210	1,147	417	156	144
	Number of girls	337	2,331	1,257	318	181	101
	Percentage	8.01%	50.56%	26.77%	8.18%	3.75%	2.73%

**Table 5:** Types of sports injuries in college physical fitness tests.

Types	Frequency order	Number of people	Percentage (%)
Strains	1	3,971	48.06
Sprains	2	3,467	41.96
Bruises	3	797	9.65
Fractures	4	27	0.33

**Table 6:** Strong rules.

Serial number	Test items	Support	Confidence
1	Pull-ups	0.002	0.814
2	Sprints	0.002	0.977
3	Long jump	0.002	0.841
4	Long run	0.002	0.756
5	Sit-ups	0.002	0.731
6	Sitting forward bending	0.001	0.678

**Table 7:** Frequency of causes of sports injuries.

Reasons	Number	Frequency of occurrence among boys	Frequency of occurrence among girls
Irregular technical actions	1	5	6
Lack of preparation	2	7	5
Inattention	3	6	7
Physical fatigue	4	4	5
Insufficient flexibility	5	3	8
Lack of self-protection	6	8	4

## Data Availability

No data were used to support this study.
